The article "WRN inhibits oxidative stress-induced apoptosis of human lensepithelial cells through ATM/p53 signaling pathway and its expression is downregulated by DNA methylation" was retracted in 2021. Reasons: errors in the materials; errors in the methods; unreliable results or conclusions.

# WRN inhibits oxidative stress-induced apoptosis of human lensepithelial cells through ATM/p53 signaling pathway and its expression is downregulated by DNA methylation

**DOI:** 10.1186/s10020-020-00187-x

**Published:** 2020-07-08

**Authors:** Shengqun Jiang, Jiansu Chen

**Affiliations:** 1 Ophthalmology Department, The First Affiliated Hospital of Jinan University Guangzhou, No.601 Huangpu Avenue West, Guangzhou, Guangdong Province China; 2 Ophthalmology Department, The First Affiliated Hospital of Bengbu Medical College, Bengbu, Anhui Province China

**Keywords:** WRN, DNA methylation, Apoptosis, Oxidative stress, ATM/p53, Age related cataract

## Abstract

**Background:**

Apoptosis and oxidative stress are the main etiology of age related cataract (ARC). This article aims to investigate the role of WRN in lens epithelial cells (LECs).

**Methods:**

We estimated the methylation level of WRN in anterior lens capsule tissues of ARC patients. SRA01/04 (LECs) cells were treated with H_2_O_2_ or combined with 5-aza-2-deoxycytidine (5-Aza-CdR) or chloroquine. CCK8 and flow cytometry were performed to explore proliferation and apoptosis. The content of ROS was detected by fluorescent probe DCFH-DA. The gene and protein expression was assessed by quantitative real-time PCR or western blot.

**Results:**

WRN was down-regulated and the methylation level of WRN was increased in the anterior lens capsule tissues. WRN overexpression and 5-Aza-CdR enhanced proliferation and repressed apoptosis and oxidative stress of SRA01/04 cells. 5-Aza-CdR enhanced WRN expression. WRN knockdown inhibited proliferation and promoted apoptosis and oxidative stress of SRA01/04 cells, which was rescued by 5-Aza-CdR. WRN overexpression and 5-Aza-CdR repressed ATM/p53 signaling pathway. Furthermore, chloroquine inhibited proliferation and promoted apoptosis and oxidative stress of SRA01/04 cells by activating ATM/p53 signaling pathway. The influence conferred by chloroquine was abolished by WRN overexpression.

**Conclusion:**

Our study reveals that DNA methylation mediated WRN inhibits apoptosis and oxidative stress of human LECs through ATM/p53 signaling pathway.

## Background

Age related cataract (ARC), also known as senile cataract, is the world’s first blind eye disease (Zhang et al. 2011). At present, surgery is still the only effective treatment for cataract. Therefore, it is urgent to study the pathogenesis of ARC and find the cause of ARC. Lens epithelial cells (LECs) are the only cleavage-active cells in the lens that can divide and differentiate into lens fiber cells and produce lens proteins. LECs play a crucial role in maintaining the stability of the lens environment and the osmotic pressure of the lens and resisting the damage of external harmful factors (Su et al. 2011; Mattioli and Thomas 2010). The occurrence of ARC is closely associated with DNA damage caused by oxidative stress in the lens (Yang et al. 2018). H_2_O_2_ induces oxidative stress in LECs by causing abnormal expression of some functional genes to cause ARC, including encoding DNA repair proteins, antioxidant defense enzymes, molecular chaperones, protein biosynthesis enzymes, and trafficking and degradation proteins (Sumanta Goswami et al. 2003; Wang et al. 2018a). Oxidative stress produces excessive reactive oxygen radicals that can damage DNA in cells. Reactive oxygen radicals convert to form hydroxyl radicals and act on DNA to cause DNA breakage, thereby resulting in apoptosis and ARC formation (Rooban et al. 2012). Oxidative stress also causes apoptosis of the LECs by causing cell membrane permeability changes, protein conformational changes, thereby resulting in lens opacity (Goswami 2003). Apoptosis of LECs is the cytological basis for the formation of all types of cataracts other than congenital cataracts (Li 1995). One study reports that oxidative damage is increased in LECs and peripheral blood lymphocytes in patients with ARC (Zhang et al. 2014).

The DNA damage repair gene, WRN, is one of the major members of the human RecQ helicase family. Many studies have shown that mutations in WRN are associated with the development of ARC. Our previous study has found that rs1346044 of WRN gene is associated with the occurrence of ARC, and the C allele has a protective effect on the occurrence of ARC. The C → T of rs1346044 leads to the mutation of the cysteine at position 1367 of the WRN gene to arginine, which increases the susceptibility of cortical ARC in Chinese Han population (Jiang et al. 2013a). The copy number variation of WRN may be related to the susceptibility of ARC in Chinese Han population, especially nuclear and posterior subcapsular ARC (Jiang et al. 2013b). Our previous study has confirms that the mRNA and protein expression levels of WRN in LECs of ARC patients are down-regulated, and the CpG islands in the promoter region of WRN gene are hypermethylated. And the protein expression of WRN is increased in lens epithelial cells (HLEB-3) after treated with methylation transferase inhibitor 5-aza-2-deoxycytidine (5-Aza-CdR) (Zhu et al. 2015). It indicates that the WRN expression in ARC is regulated by DNA methylation.

ATM protein kinase is a product encoded by the telangiectasia ataxia mutated gene ATM, which senses DNA damage, transmits DNA damage signals to downstream target genes, initiates stress systems and produces cycle arrest, cell repair and apoptosis (Berger et al. 2017). In addition, the p53 pathway plays an important role in the body response to DNA damage (Speidel 2015). The podophyllotoxin derivative XWL-1-48 triggers DNA damage by activating the ATM/p53/p21 signaling pathway (Wang et al. 2018b). Up-regulation of p53 inhibits the antioxidant capacity and cell viability of LECs, which is associated with the occurrence of ARC (Lu et al. 2018). Therefore, we hypothesized that WRN down-regulation in ARC is regulated by DNA methylation, and WRN may mediate apoptosis and oxidative damage of LECs via ATM/p53 signaling pathway.

## Materials and methods

### Collection of the anterior lens capsule tissues

A continuous annular capsulorhexis is performed on the anterior lens capsule during cataract surgery. The anterior lens capsule with a diameter of 5–5.5 mm was washed with PBS for 3 times and stored at − 80 °C. Anterior lens capsule tissues were obtained from the patients with different types of ARC (cortical, nuclear and posterior subcapsular cataract). The healthy anterior lens capsule tissues were obtained from age-matched person as control. All patients were informed and gave written consent. All protocols were authorized by the Ethics Committee of The First Affiliated Hospital of Bengbu Medical College.

### Cell culture and treatment

Human lens epithelial cell line, SRA01/04, was purchased from ATCC (Manassas, VA, USA). SRA01/04 cells were cultured in dulbecco’s modified eagle medium (DMEM) containing 10% fetal bovine serum and 1% penicillin/streptomycin in a humidified atmosphere at 37 °C and 5% CO_2_. SRA01/04 cells at exponential stage were seeded in six-well plate at a density of 1 × 10^6^ cells/mL. These cells were treated with different concentrations (0, 25, 50 and 100 μM) of H_2_O_2_ (Sangon Biotech, Shanghai, China) for 24 h. In the subsequent experiments, H_2_O_2_ at a concentration of 100 μM was used to treat cells for 24 h. After that, H_2_O_2_-induced SRA01/04 cells were treated with 10 μM 5-Aza-CdR (Sigma-Aldrich, St. Louis, MO, USA) for 72 h. 5-Aza-CdR was replaced every 24 h. SRA01/04 cells were treated with 50 μM chloroquine (ATM activator) for 24 h.

### Methylation-specific PCR (MSP)

The genome DNA of anterior lens capsule tissues was extracted using Rapid Animal Genomic DNA Isolation Kit (Sangon Biotech). The methylation of DNA samples was performed using Mag-DNA Modification Kit (Sangon Biotech). MSP was performed with the methylated DNA as template. The primers set specific to methylated DNA and un-methylated DNA were purchased from Sangon Biotech.

### Cell transfection

Plasmid vector pcDNA3.1-WRN and its negative control (pcDNA3.1-NC) were constructed by RIBOBIO (Shanghai, China) via standard molecular cloning approaches. Small interfering RNA (siRNA) specific targeting WRN (WRN siRNA) and the corresponding NC (Scramble) were purchased from RIBOBIO. These vectors were transfected into SRA01/04 cells separately. The cell transfection assay was performed using Lipofectamine 2000 Transfection Reagent (Invitrogen, Carlsbad, CA, USA) according to the manufacturer’s protocol.

### Quantitative real-time PCR (qRT-PCR)

QRT-PCR was performed to measure the expression intensity of different genes. Total RNA was extracted from anterior lens capsule tissues or SRA01/04 cells using RNAprep Pure Tissue Kit (Tiangen, Beijing, China). The purity and concentration of RNA was detected using a NanoDrop 2000 spectrophotometer (Thermo Fisher Scientific, Waltham, MA, USA). The RNA was converted to complementary DNA using PrimeScript™ RT Reagent Kit (Takara, Tokyo, Japan). QRT-PCR was carried out using SYBR Green PCR Mix Kit (Takara) according to the instruction. The results were analyzed using the ∆∆CT (cycle threshold) method for quantification.

### Western blot (WB)

The total protein was extracted from anterior lens capsule tissues or SRA01/04 cells using Tissue or Cell Total Protein Extraction Kit (Sangon Biotech). Equivalent protein from different samples were separated by protein electrophoresis and transferred on PVDF membranes. The membranes were incubated with antibodies against the test proteins after treated with sealed liquid. After the membranes were washed with TBST for several times, secondary antibodies labeled with horseradish peroxidase were incubated with the membranes. GAPDH or β-actin was used as a reference protein for normalization. The gray level of the protein bands was examined by Image J software.

### Cell viability

The CCK8 assay was performed to explore the proliferation ability of SRA01/04 cells. The cells were treated with pancreatin after the cell density reached 80%. The cells were then re-suspended in DMEM containing 10% fetal bovine serum and the cell density was adjusted to 1 × 10^5^/mL. The cell suspension (100 μL) and CCK8 reagent (10 μL) were mixed and seeded into 96-well plates. Then, the cells were cultured in an incubator at 37 °C for 4 h. The optical density of samples was detected at 450 nm wavelength using enzyme-labeled instrument (Thermo Fisher Scientific).

### Cell apoptosis

The cells were collected by centrifuging for 5 min at the speed of 500×g, 4 °C. The cells were washed with pre-cooling PBS for 2 times. Cells were then resuspended in the Annexin V Binding buffer. The cell suspension was dyed with Annexin V-FITC and PI and plunged into darkness at room temperature for 15 min. Then, the cell suspension was mixed with Annexin V Binding buffer and put on ice. The apoptosis rate of cells was determined by flow cytometry in an hour. The assay was performed according to the instruction of Annexin V-FITC/PI Cell Apoptosis Detection Kit (TransGen Biotech, Beijing, China).

### Detection of intracellular reactive oxygen species (ROS)

SRA01/04 cells were seeded into 24-well plate and cultured for 24 h. After centrifugation the supernatant was discarded. The cells was resuspended in 1 mL DCFH-DA (10 μM) and incubated in an incubator at 37 °C for 20 min. The cells are mixed every 5 min. The cells were washed with serum-free DMEM for 3 times. The fluorescence intensity of the cells was observed by confocal laser scanning microscope (LEICA, Wetzlar, Germany). Detection conditions: excitation wavelength 488 nm, emission wavelength 525 nm, and the grating width of the excitation and emission wavelengths is 5 nm. The assay was performed according to the instruction of Reactive Oxygen Species Assay Kit (Solarbio, Beijing, China).

### Statistical analysis

All experiments were independently repeated at least 3 times. All values were exhibited as mean ± standard deviation and analyzed by SPSS 22.0 statistical software (IBM, Armonk, NY, USA). For comparison of two groups, a two-tailed Student’s t test was used. Comparison of multiple groups was made using a one- or two-way ANOVA. *P* < 0.05 was considered statistically significant.

## Results

### The expression of WRN is decreased and the methylation level of WRN is increased in the anterior lens capsule tissues of patients with ARC

To investigate the involvement of WRN in ARC, we analyzed its expression and methylation level in the anterior lens capsule tissues of patients with different types of ARC (cortical, nuclear and posterior subcapsular cataract). Compared with the healthy anterior lens capsule tissues of age-matched person, the gene and protein expression of WRN was significantly reduced in the three types of diseased anterior lens capsule tissues (Fig. 1a and b). And the methylation level of WRN was higher in the three types of diseased anterior lens capsule tissues than that in the healthy anterior lens capsule tissues (Fig. 1c).

**Fig. 1:** The expression of WRN is decreased and the methylation level of WRN is increased in the anterior lens capsule tissues of patients with ARC. Anterior lens capsule tissues were obtained from the patients with different types of ARC (cortical, nuclear and posterior subcapsular cataract). The healthy anterior lens capsule tissues from age-matched person were as control. **a** QRT-PCR and **b** WB were performed to detect the gene and protein expression of WRN in the anterior lens capsule tissues. **c** MSP was performed to detect the methylation level of WRN in the anterior lens capsule tissues. M: methylation; U: unmethylation. (^**^P < 0.01 compared with the Control group)

### WRN overexpression suppresses apoptosis and oxidative stress of SRA01/04 cells in vitro

In order to define the role of WRN in the anterior lens capsule tissues, we detected the expression and methylation level of WRN in SRA01/04 cells after treated with different concentrations of H_2_O_2_. The gene and protein expression level of WRN was gradually decreased with the increase of H_2_O_2_ concentration (Fig. 2a and b). The methylation level of WRN was gradually increased with the increase of H_2_O_2_ concentration (Fig. 2c). And H_2_O_2_ at a concentration of 100 μM had the greatest influence on the expression and methylation level of WRN in SRA01/04 cells. Therefore, in the subsequent experiments, H_2_O_2_ at a concentration of 100 μM was used to treat the SRA01/04 cells. In addition, WRN was up-regulated in SRA01/04 cells, and then the modified SRA01/04 cells were treated with 100 μM H_2_O_2_. CCK8 assay and flow cytometry were assessed cell proliferation and apoptosis of SRA01/04 cells. H_2_O_2_ treatment led to a decrease in cell proliferation of SRA01/04 cells, which was effectively rescued by WRN overexpression (Fig. 2d). H_2_O_2_ treatment markedly facilitated apoptosis of SRA01/04 cells, and its promoting effect on apoptosis was dramatically reduced by WRN overexpression (Fig. 2e). In addition, the level of ROS and malondialdehyde (MDA) was significantly increased in SRA01/04 cells after H_2_O_2_ treatment, and significantly decreased in SRA01/04 cells after transfected with pcDNA3.1-WRN (Fig. 2f and g). On the contrary, H_2_O_2_-treated SRA01/04 cells exhibited a decrease in the expression of superoxide dismutase (SOD) and catalase (CAT), and WRN overexpression promoted the expression of SOD and CAT in SRA01/04 cells (Fig. 2g). These results taken together reveal that WRN overexpression suppressed apoptosis and oxidative stress and promoted cell proliferation of SRA01/04 cells in vitro.

**Fig. 2:** WRN overexpression suppresses apoptosis and oxidative stress of SRA01/04 cells in vitro. SRA01/04 cells were treated with different concentrations (0, 25, 50 and 100 μM) of H_2_O_2_. **a** QRT-PCR and (**b**) WB were performed to estimate the gene and protein expression of WRN in the SRA01/04 cells. **c** MSP was performed to detect the methylation level of WRN in the SRA01/04 cells. SRA01/04 cells were transfected with pcDNA3.1-WRN or pcDNA3.1-NC, and then the modified SRA01/04 cells were treated with 100 μM H_2_O_2_. **d** CCK8 was performed to explore the cell proliferation of the modified SRA01/04 cells. **e** The apoptosis of the modified SRA01/04 cells was determined by flow cytometry. **f** The content of ROS in the modified SRA01/04 cells was detected by fluorescent probe DCFH-DA. **g** WB was performed to detect the expression of SOD, CAT and MDA in the modified SRA01/04 cells. M: methylation; U: unmethylation. (^*^P < 0.05 compared with the 0 μM H_2_O_2_ or Control group, ^**^P < 0.01 compared with the 0 μM H_2_O_2_ or Control group, ^#^*P* < 0.05 compared with the H_2_O_2_ + Vector group, ^##^*P* < 0.01 compared with the H_2_O_2_ + Vector group)

### 5-Aza-CdR treatment suppresses apoptosis and oxidative stress of SRA01/04 cells in vitro

To explore the effect of 5-Aza-CdR on apoptosis and oxidative stress of SRA01/04 cells, H_2_O_2_-induced SRA01/04 cells were treated with 5-Aza-CdR. We found that the gene and protein expression of WRN were obviously reduced in H_2_O_2_-induced SRA01/04 cells, which was effectively abolished by 5-Aza-CdR treatment (Fig. 3a and b). Furthermore, we performed CCK8 assay and flow cytometry to examine cell proliferation and apoptosis of SRA01/04 cells. The cell proliferation was lower in SRA01/04 cells after H_2_O_2_ treatment than that in normal SRA01/04 cells. 5-Aza-CdR-treated SRA01/04 cells exhibited an increase in cell proliferation (Fig. 3c). The apoptosis was markedly promoted by H_2_O_2_ treatment and repressed by 5-Aza-CdR treatment in SRA01/04 cells (Fig. 3d). In addition, the level of ROS, SOD, CAT and MDA in the SRA01/04 cells were detected by fluorescent probe DCFH-DA and WB. As shown in Fig. 3e and f, the level of ROS and MDA were significantly increased in SRA01/04 cells after H_2_O_2_ treatment, and significantly decreased in SRA01/04 cells after treated with 5-Aza-CdR and H_2_O_2_. On the contrary, H_2_O_2_ treatment inhibited the expression of SOD and CAT in SRA01/04 cells. And the influence conferred by H_2_O_2_ treatment was abolished by 5-Aza-CdR (Fig. 3f). These data suggest that 5-Aza-CdR treatment inhibits apoptosis and oxidative stress and promotes cell proliferation of SRA01/04 cells in vitro.

**Fig. 3:** 5-Aza-CdR treatment suppresses apoptosis and oxidative stress of SRA01/04 cells in vitro. SRA01/04 cells were consecutively treated with 100 μM H_2_O_2_ and 5-Aza-CdR. Normal SRA01/04 cells served as control. **a** QRT-PCR and (**b**) WB were performed to detect the gene and protein expression of WRN in the SRA01/04 cells. **c** CCK8 was performed to explore the cell proliferation of the SRA01/04 cells. **d** The apoptosis of the SRA01/04 cells was determined by flow cytometry. **e** The content of ROS in the SRA01/04 cells was detected by fluorescent probe DCFH-DA. **f** WB was performed to explore the expression of SOD, CAT and MDA in the SRA01/04 cells. (^**^P < 0.01 compared with the Control group, ^##^*P* < 0.01 compared with the H_2_O_2_ group)

### 5-Aza-CdR treatment suppresses apoptosis and oxidative stress of SRA01/04 cells by promoting WRN expression in vitro

To further investigate the molecular mechanism of 5-Aza-CdR in regulating apoptosis and oxidative stress of SRA01/04 cells, we silenced WRN in SRA01/04 cells. Then, we performed qRT-PCR and WB to estimate the gene and protein expression of WRN in the SRA01/04 cells. We found that WRN silencing led to a decrease in the gene and protein expression of WRN in the SRA01/04 cells (Fig. 4a and b). Furthermore, the normal and modified SRA01/04 cells were consecutively treated with H_2_O_2_ and 5-Aza-CdR. The gene and protein expression of WRN in the SRA01/04 cells was notably enhanced by 5-Aza-CdR. WRN-silenced SRA01/04 cells exhibited a decrease in the gene and protein expression of WRN, which was effectively recused by 5-Aza-CdR (Fig. 4c and d). Moreover, the cell proliferation and apoptosis of SRA01/04 cells were estimated by CCK8 assay and flow cytometry. 5-Aza-CdR significantly promoted cell proliferation of SRA01/04 cells, whereas WRN knockdown severely repressed apoptosis of SRA01/04 cells. The inhibiting effect of WRN down-regulation on cell proliferation of SRA01/04 cells was rescued by 5-Aza-CdR (Fig. 4e). The apoptosis of SRA01/04 cells was repressed by 5-Aza-CdR and enhanced by WRN silencing. WRN-silenced SRA01/04 cells displayed an increase in apoptosis after 5-Aza-CdR treatment (Fig. 4f). In addition, the content of ROS and the expression of SOD, CAT and MDA in the SRA01/04 cells were detected by fluorescent probe DCFH-DA and WB. Figure 4g and h show that the level of ROS and MDA in the SRA01/04 cells was suppressed by 5-Aza-CdR and enhanced by WRN silencing. The influence conferred by WRN silencing was abolished by 5-Aza-CdR treatment. 5-Aza-CdR caused a boost in the levels of SOD and CAT in the SRA01/04 cells. And WRN-silenced SRA01/04 cells exhibited a decrease in the level of SOD and CAT, which was effectively rescued by 5-Aza-CdR treatment (Fig. 4h). Therefore, these findings confirm that 5-Aza-CdR treatment suppresses apoptosis and oxidative stress of SRA01/04 cells by promoting WRN expression in vitro.

**Fig. 4:** 5-Aza-CdR treatment suppresses apoptosis and oxidative stress of SRA01/04 cells by promoting WRN expression in vitro. SRA01/04 cells were transfected with WRN siRNA or Scramble. Normal SRA01/04 cells served as control. **a** QRT-PCR and (**b**) WB were performed to detect the gene and protein expression of WRN in the modified SRA01/04 cells. The normal and modified SRA01/04 cells were consecutively treated with 100 μM H_2_O_2_ and 5-Aza-CdR. **c** QRT-PCR and **d** WB were performed to detect the gene and protein expression of WRN in the modified SRA01/04 cells. **e** CCK8 was performed to explore the cell proliferation of the modified SRA01/04 cells. **f** The apoptosis of the modified SRA01/04 cells was determined by flow cytometry. **g** The content of ROS in the modified SRA01/04 cells was detected by fluorescent probe DCFH-DA. **h** WB was performed to detect the expression of SOD, CAT and MDA in the modified SRA01/04 cells. (^**^P < 0.01 compared with the Scramble group, ^##^*P* < 0.01 compared with the Control or Control+Scramble group, ^$$^*P* < 0.01 compared with the Control+WRN siRNA group)

### WRN overexpression inhibits ATM/p53 signaling pathway

To investigate whether WRN overexpression has an inhibiting effect on ATM/p53 signal pathway, we detected the effect of WRN overexpression and 5-Aza-CdR treatment on the expression of ATM/p53 signaling pathway-related proteins in SRA01/04 cells by WB. As shown in Fig. 5a and b, H_2_O_2_ treatment had no effect on ATM expression in SRA01/04 cells. And H_2_O_2_ treatment significantly promoted the expression of p-ATM, p53, p-p53, p21, Bax, PUMA and NOXA in SRA01/04 cells. WRN overexpression and 5-Aza-CdR treatment had on effect on the expression of ATM in SRA01/04 cells. However, WRN overexpression and 5-Aza-CdR treatment obviously suppressed the expression of p-ATM, p53, p-p53, p21, Bax, PUMA and NOXA in SRA01/04 cells (Fig. 5a and b). These data show that WRN overexpression inhibits ATM/p53 signaling pathway.

**Fig. 5:** WRN overexpression inhibits ATM/p53 signaling pathway. SRA01/04 cells were transfected with pcDNA3.1-WRN or pcDNA3.1-NC, and then the modified SRA01/04 cells were treated with 100 μM H_2_O_2_. **a** WB was performed to detect the expression of p-ATM, ATM, p53, p-p53, p21, Bax, PUMA and NOXA in the modified SRA01/04 cells. SRA01/04 cells were consecutively treated with 100 μM H_2_O_2_ and 5-Aza-CdR. **b** WB was performed to estimate the expression of p-ATM, ATM, p53, p-p53, p21, Bax, PUMA and NOXA in the modified SRA01/04 cells.(^**^P < 0.01 compared with the Control group, ^##^*P* < 0.01 compared with the H_2_O_2_ + Vector group, ^$^*P* < 0.05 compared with the H_2_O_2_ group, ^$$^*P* < 0.01 compared with the H_2_O_2_ group)

### WRN overexpression inhibits apoptosis and oxidative stress of SRA01/04 cells via ATM/p53 signaling pathway

To explore the molecular mechanism of WRN in ARC, SRA01/04 cells were treated with chloroquine to activate ATM/p53 signaling pathway. As shown in Fig. 6a, WRN overexpression and chloroquine treatment had no effect on ATM expression in SRA01/04 cells. WRN overexpression apparently inhibited the expression of p-ATM, p53, p-p53, p21, Bax, PUMA and NOXA, and chloroquine treatment distinctly promoted the expression of p-ATM, p53, p-p53, p21, Bax, PUMA and NOXA in SRA01/04 cells. And the promoting effect of chloroquine treatment on the expression of p-ATM, p53, p-p53, p21, Bax, PUMA and NOXA in SRA01/04 cells was rescued by WRN overexpression (Fig. 6a). WRN overexpression caused an increase in cell proliferation, and chloroquine treatment led to a decrease in cell proliferation in SRA01/04 cells. The influence conferred by chloroquine treatment was abolished by WRN overexpression (Fig. 6b). Apoptosis was lower in SRA01/04 cells after transfected with pcDNA3.1-WRN than that in the noraml SRA01/04 cells. Chloroquine-treated SRA01/04 cells displayed a boost in apoptosis, which was effectively abolished by WRN up-regulation (Fig. 6c). As shown in Fig. 6d and e, the levels of ROS and MDA were significantly decreased in SRA01/04 cells after transfected with pcDNA3.1-WRN, and distinctly increased in SRA01/04 cells after chloroquine treatment. WRN up-regulation markedly inhibited the promoting effect of chloroquine treatment on the levels of ROS and MDA in SRA01/04 cells. On the contrary, WRN up-regulation promoted the expression of SOD and CAT, and chloroquine treatment inhibited the expression of SOD and CAT in SRA01/04 cells. And the inhibiting effect of chloroquine treatment on the expression of SOD and CAT in SRA01/04 cells was rescued by WRN overexpression (Fig. 6e). Therefore, these data indicate that WRN overexpression inhibits apoptosis and oxidative stress of SRA01/04 cells via ATM/p53 signaling pathway.

**Fig. 6:** WRN overexpression inhibits apoptosis and oxidative stress of SRA01/04 cells via ATM/p53 signaling pathway. SRA01/04 cells were transfected with pcDNA3.1-WRN or pcDNA3.1-NC, and then the modified SRA01/04 cells were treated with 50 μM chloroquine. **a** WB was performed to detect the expression of p-ATM, ATM, p53, p-p53, p21, Bax, PUMA and NOXA in the modified SRA01/04 cells. **b** CCK8 was performed to explore the cell proliferation of the modified SRA01/04 cells. **c** The apoptosis of the modified SRA01/04 cells was determined by flow cytometry. **d** The content of ROS in the modified SRA01/04 cells was detected by fluorescent probe DCFH-DA. **e** WB was performed to explore the expression of SOD, CAT and MDA in the modified SRA01/04 cells. (^*^P < 0.05 compared with the Vector group, ^**^P < 0.01 compared with the Vector group, ^#^*P* < 0.05 compared with the Vector+Chl group, ^##^*P* < 0.01 compared with the Vector+Chl group)

## Discussion

ARC is a common disease in the elderly and is one of the phenomena of human aging. As the age increases, the intraocular lens will slowly harden, turbid, and affect vision. The LECs play a vital role in the growth and development of lens and in maintaining the transparency and stability of the lens (Mccarty 2001). Pathological changes in LECs will inevitably lead to lens lesions, such as the occurrence of cataracts and the development of posterior cataracts (Zhang et al. 2002). A series of degenerative changes occurs in LECs during the formation of cataracts, in which the apoptosis of LECs participates in this process. In addition, oxidative stress is a common pathway for the occurrence of ARC caused by various external factors (Goswami 2003). With the increase of age, the content of antioxidants such as glutathione in the human lens gradually decreases, and the ability to scavenge oxygen free radicals gradually decreases. The denaturation and aggregation of lens proteins caused by oxidative damage leads to the increase of lens scattering, thereby resulting in opacity of the lens and the occurrence of ARC. But the molecular mechanisms of apoptosis and oxidative stress in human lens epithelial cells remain unknown. Our previous study has found that WRN gene is closely associated with the occurrence of ARC (Jiang et al. 2013a). In our study, we further explored the effect of WRN expression on apoptosis and oxidative stress in LECs of ARC. Our data showed that the expression of WRN is remarkably decreased and the methylation level of WRN is significantly increased in the anterior lens capsule tissues of patients with ARC.

Studies have found that hypermethylation of the WRN promoter region results in low expression of WRN protein in tumor tissues and increases chromosome instability in a variety of tumors. WRN shows the characteristics of inhibiting tumors (Agrelo et al. 2006). On the other hand, low expression of the WRN protein promotes the sensitivity of tumor cells to chemotherapeutic drugs (topological enzyme inhibition). The detection of methylation in the WRN promoter region in tumor tissues provides a good basis for screening patients who are suitable for chemotherapy drugs (Masuda et al. 2012; Wang and Wang 2013). Many studies also have shown that WRN is closely associated with apoptosis. In microsatellite instability models, WRN knock-out induces double-stranded DNA breaks and promotes apoptosis and cell cycle arrest selectively (Chan et al. 2019). The Werner syndrome ATP-dependent helicase encoded by WRN gene is closely related to cell proliferation and DNA repair. The cell cycle arrest and apoptosis is obviously induced in human T-cell leukemia virus type 1-transformed leukemia cells after treated by WRN inhibitor (NSC 19630) (Moles et al. 2016). In our study, H_2_O_2_ treatment inhibited the expression of WRN and promoted the methylation level of WRN in SRA01/04 cells. H_2_O_2_ treatment led to a decrease of cell proliferation and caused an increase of apoptosis in SRA01/04 cells. H_2_O_2_-treated SRA01/04 cells exhibited a boost in the levels of ROS and MDA, and a decrease in the levels of SOD and CAT. SOD2 is one of the endogenous antioxidant enzymes that protect against reactive oxygen species. Previous study has confirmed that H_2_O_2_ induces the up-regulation of miR-146a, which interacts with SOD2 and inhibits the expression of SOD2 (Ji et al. 2013). H_2_O_2_ treatment promotes the generation of excess ROS, which then causes MDA formation, thereby resulting in cell death (Xia et al. 2018). Thus, these findings indicate that H_2_O_2_ treatment induces apoptosis and oxidative stress, and represses cell proliferation of SRA01/04 cells. In addition, the influence conferred by H_2_O_2_ treatment was rescued by WRN overexpression. Furthermore, 5-Aza-CdR treatment significantly promoted the expression of WRN. And 5-Aza-CdR treatment enhanced cell proliferation, suppressed apoptosis and oxidative stress in SRA01/04 cells. WRN silencing caused a decrease in cell proliferation, and led to an increase in apoptosis and oxidative stress in SRA01/04 cells, which was effectively rescued by 5-Aza-CdR treatment. Therefore, these data taken together reveal that 5-Aza-CdR treatment inhibits apoptosis and oxidative stress and promotes cell proliferation of SRA01/04 cells by up-regulating WRN expression.

One study shows that the ATM/p53/p21 signaling pathway induces G2/M arrest and mediates DNA damage (Li et al. 2018). Under DNA damage conditions, activated ATM kinase phosphorylates p53 and drives cell senescence or apoptosis. Phosphorylation of p53 is the first step in initiating oxidative stress response. Activation of p53 protein activates cell cycle checkpoint p21 expression, thereby inhibiting cell cycle and repairing damaged DNA. Apoptosis occurs when DNA repair fails. Our research found that WRN overexpression and 5-Aza-CdR treatment inhibited the expression of p-ATM, p53, p-p53 and p21 in the SRA01/04. And the expression of PUMA, NOXA and Bax was notably repressed by WRN overexpression and 5-Aza-CdR treatment. PUMA and NOXA were the target gene of pro-apoptotic p53. It indicates that WRN overexpression and 5-Aza-CdR treatment inhibits apoptosis via ATM/p53 signaling pathway. Moreover, chloroquine was used to induce ATM activation. Chromatin and chromosome structures can be altered in the absence of DNA breaks by exposure to chloroquine. Then, the changes in chromatin structure lead to ATM activation (Bakkenist and MB K. 2003). We found that chloroquine treatment inhibited cell proliferation, and enhanced apoptosis and oxidative stress by activating ATM/p53 signaling pathway, which was effectively abolished by WRN up-regulation.

## Conclusions

In conclusion, our study demonstrates that DNA methylation mediated WRN inhibits apoptosis and oxidative stress of human LECs via ATM/p53 singling pathway. The results imply that WRN might play certain roles in the pathogenesis of ARC and supply the new target point and strategy for the treatment of ARC.

## Data Availability

The datasets used and/or analysed during the current study are available from the corresponding author on reasonable request.

## Abbreviations

5-Aza-CdR: 5-aza-2-deoxycytidine
ARC: Age related cataract
CAT: Catalase
DMEM: Dulbecco’s modified eagle medium
LECs: Lens epithelial cells
MDA: Malondialdehyde
MSP: Methylation-Specific PCR
qRT-PCR: Quantitative real-time PCR
SOD: Superoxide dismutase
WB: Western blot
